# A Novel Developed Bioactive Composite Resin Containing Silver/Zinc Oxide (Ag/ZnO) Nanoparticles as an Antimicrobial Material against *Streptococcus mutans*, *Lactobacillus*, and *Candida albicans*

**DOI:** 10.1155/2021/4743411

**Published:** 2021-10-16

**Authors:** Mojgan Kachoei, Baharak Divband, Mahdi Rahbar, Mahdiyeh Esmaeilzadeh, Milad Ghanizadeh, Mostafa Alam

**Affiliations:** ^1^Department of Orthodontics, Faculty of Dentistry, Tabriz University of Medical Sciences, Tabriz, Iran; ^2^Dental and Periodontal Research Center, Faculty of Dentistry, Tabriz University of Medical Sciences, Tabriz, Iran; ^3^Department of Inorganic Chemistry, Faculty of Chemistry, University of Tabriz, Tabriz, Iran; ^4^Department of Esthetic and Restorative Dentistry, School of Dentistry, Ardabil University of Medical Sciences, Ardabil, Iran; ^5^Student Research Committee, Faculty of Dentistry, Tabriz University of Medical Sciences, Tabriz, Iran; ^6^Oral and Maxillofacial Surgery Department, Faculty of Dentistry, Tabriz University of Medical Sciences, Tabriz, Iran; ^7^Department of Oral and Maxillofacial Surgery, School of Dentistry, Shahid Beheshti University of Medical Sciences, Tehran, Iran

## Abstract

**Aim:**

The objectives of this study were to develop a new bioactive composite resin containing silver/zinc oxide (Ag/ZnO) nanoparticles and investigate the effects on mechanical, cytotoxic, biocompatibility, and antimicrobial properties.

**Materials and Methods:**

Disc-shaped specimens were prepared from composite with and without nanoparticles in separate culture media containing *Streptococcus mutans*, *Lactobacillus*, and *Candida albicans*. Bracket bonding evaluation was performed on composite without nanoparticles (O), composite containing ZnO (Z) nanoparticles, composite containing ZnO nanoparticles and silver ions (A&Z), and composite containing Ag/ZnO nanoparticles (AZ) synthesized using optical precipitation.

**Results:**

Composite resin with nanoparticles (AZ, A&Z, and Z) showed significant antimicrobial properties (*P* < 0.05). The mean shear bond strength of A&Z composite resin (13.61 ± 0.73 MPa) was significantly less than that of conventional composite resin (19.03 ± 4.12 MPa) (*P* < 0.05). In addition, the mean shear bond strength of AZ composite resin (20.49 ± 1.03 MPa) was significantly higher than that of Z (16.35 ± 1.03 MPa) and A&Z composite resins.

**Conclusions:**

Incorporation of ZnO nanoparticles and their compounds into orthodontic composite resins induced antibacterial properties against oral pathogens, and of all these nanoparticles, the AZ group exhibited the best antimicrobial activity and highest shear bond strength.

## 1. Introduction

Orthodontic treatment possesses many advantages for patients with functional and esthetic problems and results in the satisfaction of the majority of such patients. However, such treatment might have complications for these patients, including demineralization, caries, and tooth discoloration around brackets and the bonded areas in the form of white spot lesions (WSL), which are considered a major challenge for clinicians and a major challenge factor for dissatisfaction of patients. This problem makes the patients susceptible to more widespread caries, especially in patients with poor oral hygiene. In this context, patients receiving a full fixed treatment plan are more susceptible to caries and exhibit a significant increase in *S. mutans* counts in their plaque and saliva [1, 2]. In the presence of an increased count of cariogenic bacteria in the saliva and plaque and poor oral hygiene, decalcification and carious lesions can occur in less than 4 weeks [3, 4].

Fluoride-containing materials, especially fluoride varnishes, are widely used to prevent caries. Still, they have two main problems: first, they need regular patient cooperation, and second, they have a moderate effect on prevention of WSL and caries [5]. Fluoride-containing bonding agents as well have the problem of rapid release during the first 24 hours, with a decrease in release over time [2]. Nanoparticles (NPs) have been broadly used as antimicrobial agents in medicine and dentistry. Nanoparticles are particles smaller than 100 nm in size [6]. Because of the greater surface-to-volume ratio, nanoparticles interact more closely with microbial membranes and present a considerably larger surface area for antimicrobial activity [7]. ZnO and ZnO-containing materials have significant antibacterial and antifungal activity and are used in different ways for the treatment of traumatic injuries, foot injuries, and burns [8]. Dental materials, including endodontic sealers and adhesive cements, use this property of ZnO for bonding of fixed restorations. The results of a study by Tavassoli Hojati et al. in relation to the effect of incorporating ZnO nanoparticles into flowable composite resins on the antibacterial, physical, and strength properties showed that an increase in the concentration of these nanoparticles resulted in a significant increase in the antibacterial properties of these composite resins [9].

Also, Ahn et al. improved the antibacterial properties of orthodontic composite resins as adhesive agents by adding silver nanoparticles to their structure. However, there was no significant difference between these experimental composite resins and the conventional composite resin in shear bond strength [10]. Although silver nanoparticles induce favorable antibacterial properties, they might result in a dark color in composite resin, creating esthetic problems. Ag/ZnO (AZ) nanoparticles are white, and incorporating them into composite resins with the same color does not lead to esthetic problems. On the other hand, it is expected that the use of these nanoparticles, which contain both silver and zinc oxide, will increase their antibacterial properties [10].

Application of low or nontoxic dental materials is essential in long-term usage to guarantee patient and staff health and safety. Biocompatible materials are compatible with pulp and other live tissues with minimal cytotoxic impacts [11].

Previous studies have confirmed that ZnO nanoparticles are safe and biocompatible and can be used in dental and medical applications [12]. Moreover, based on previous investigations, silver NPs showed a biocompatible behavior, which means not affecting cell metabolism and proliferation, or cause genotoxic damage to cells [7].

Considering the properties mentioned for AZ nanoparticles and the unfavorable properties of silver nanoparticles alone and since fixed orthodontic treatment requires a biocompatible material with antibacterial properties concomitant with preservation of mechanical properties, the present study was undertaken to evaluate the effect of incorporating ZnO and AZ nanoparticles into orthodontic composite resins on the antibacterial properties, biocompatibility, and shear bond strength of these composite resins for the first time.

## 2. Materials and Methods

### 2.1. Preparation of Nanoparticles

Zinc acetylacetonate, sodium hydroxide, AgNO_3_, ethanol (absolute), and starch were purchased from Merck Company (Darmstadt, Germany). As described in our previous work [13], ZnO and Ag/ZnO nanoparticles were synthesized and named as Z and AZ. As a sample, 0.4 g zinc acetylacetonate was dissolved in 20 ml absolute ethanol and 20 ml of starch solution (30%) was added drop wise, and the mixture was kept stirring for 4 h. Then, the aqueous solution of AgNO_3_ was dropped into the solution under stirring for 30 minutes and at last heated in a water bath. During the whole process, the system was continuously stirred. The solution gradually became milky gel with temperature rising up to 80°C. At last, the gel was dried at 100°C for 24 h, heated in a laboratory furnace at 400°C for 8 h to burn out the starch residues, and calcined at 550°C for 5 h. After synthesis of ZnO nanoparticles, the solution of AgNO_3_ (0.2 *µ*L) was added drop wise in the aqueous suspension of ZnO nanoparticles and named as A&Z.

Nanoparticles were mixed continuously with no-mix self-cure composite resin (Unite Bonding System; Reliance, USA) using a plastic spatula for 15 min at different concentrations of 0% (without nanoparticle), 5%, 10%, 15%, and 20% in weight. The samples were prepared in glass containers of 10 mm diameter and 1.5 mm height. An activator primer liquid was placed on the samples, and their setting time was completed. After that, the samples were polished with 600, 800, and 1200 grit SiC papers (991A Softlex, Berlin, Germany) to obtain highly polished samples with identical surface roughness (Ra) values. To confirm the Ra was homogenous, two samples from each group were observed randomly by microscope-assisted precision (MAP).

X-ray diffraction technique (XRD; Siemens D5000, Germany) was utilized in order to characterize the crystalline structure of Ag-doped ZnO nanoparticles. X-ray diffraction patterns (XRD) were collected using a Siemens D500 diffractometer with Cu k*α* radiation (=1.5418 Å and 2*θ* = 4–80°) at room temperature. A scanning electron microscope (Philips XL30) equipped with energy dispersive X-ray (EDX) facility was used to capture SEM images and to perform elemental analysis. The SEM sample was gold coated prior to examination, and SEM was operated at 5 kV while EDX analysis was performed at 15 kV. The TEM study was carried out on a Zeiss LEO 912 Omega instrument, operating at 100 kV.

### 2.2. Shear Bond Strength (SBS) Test

Different resin composites were prepared in four separate experimental groups. In group 1, composite resin was used for bonding of brackets without nanoparticles (O). In groups 2–4, composite resin with ZnO nanoparticles (Z), composite resin with ZnO nanoparticles and silver ions (A&Z), and composite resin with Ag/ZnO nanoparticles (AZ) were synthesized, respectively. The powder of nanoparticles was added to the no-mix self-cure composite resin and consistently mixed for 15 minutes by means of a glass spatula.

120 extracted human maxillary first premolars were stored in 0.01% thymol solution (Thymol Mylan, Seiyaku, Japan) at 4°C to prevent bacterial growth and dehydration. The specimens were embedded in a self-cure acrylic (Ivoclar Vivadent, Naturno BZ, Italy) block up to cementoenamel junction in a way that the labial surface of tooth vertically crossed the horizontal line of block base and were stored in distilled water at 37°C for 24 h. They were then coded from 1 to 120 (*n* = 30).

The teeth surface was cleaned with fluoride-free pumice paste using a nylon brush attached to the low-speed handpiece for 5 seconds and washed for 10 seconds by running water. The midcoronal enamel surface was etched with 37% phosphoric acid (3M Unitek, Monrovia, USA) according to manufacturer's instruction and then was thoroughly washed by water spray for 15 seconds. The excess water was removed by gentle air flow from 2 cm distance for 10 seconds. When the white chalky surface of enamel was observed, a thin layer of autopolymerization adhesive (Unite Bonding System; Reliance, USA) was applied on etched section of teeth and bracket base (ortho-organizer, stainless steel). Finally, no-mix self-cure composite (Unite Bonding System; Reliance, USA) was applied to bracket base, which was seated by the application of moderate compressive force for 10 seconds in order to obtain smooth steady composite thickness on the enamel surface.

The blocks were placed in the Hounsfield Test Equipment (Surrey, UK) and fixed in lower grip of the machine. A steel rod with the cutting edge of 0.5 mm was attached to the crosshead of the machine. Each tooth labial surface was oriented to be parallel to the force during the SBS test. The tooth placement in the machine was examined by two operators. An occlusogingival load was applied to the bracket, producing a shear force at the bracket-tooth interface. The force was measured in Newton at a crosshead speed of 0.5 mm/min and divided by the surface area of the brackets pad to calculate the SBS in megapascals (MPa).

### 2.3. Zn and Ag Release

Composite discs containing nanoparticles (5 mm × 1 mm, *n* = 5) were prepared and stored at a dry place at 37°C for 24 hours. Then, they had been separately immersed in artificial saliva (Nik Ceram Razi corporation, Isfahan, Iran) buffered at a pH of 7 using HEPES (4-(2-hydroxyethyl) piperazine-1-ethane-sulfonic acid)) solution (50 mmol/L) with a constant ratio of 3 mm^3^/mL between specimen volume and immersion medium. Specimens were kept immersed for a total of 30 days, and every 7 days, the immersing solution was totally replaced. The solutions were analyzed by inductively coupled plasma optical emission spectrometry (ICP-OEP, 700, Agilent Technologies, Santa Clara, CA, USA) to determine Zn and Ag ionic concentrations released from the composite.

### 2.4. Antibacterial Activity Assay

Antimicrobial activity of the components was investigated by using the microbroth dilution (MIC) method. In this regard, *S. mutans* ATCC 35668*, Staphylococcus aureus* ATCC 25923, *Lactobacillus gasseri* ATCC 33323, *Escherichia coli* ATCC 25922, *and Candida albicans* ATCC 10231 as common pathogens were selected and purchased from Persian microbial collection (PTCC) related to the National Research Center for Science and Technology, Tehran, Iran. For MIC identification of components, all pathogens were cultured in Mueller-Hinton agar (Merck, Germany) overnight at 37°C (for 24 hours), and yeasts were cultured in Mueller-Hinton agar plus 1% glucose under aerobic condition. Exponential growth phase of pathogens was provided by culture in Mueller-Hinton broth (Merck, Germany) at 37°C, and a concentration equal to 0.5 McFarland of the pathogens was used for study. MIC experience was done according to Clinical Laboratory Standard Institute (CLSI) protocol for microbroth dilution in 98-well polystyrene plates. Composite resins with different concentrations were exposed with pathogens. For anaerobic experience, GasPak Grade A (Merck, Germany) was used. Test groups included nanocomposite resin with different concentrations of silver and zinc oxide nanoparticles, namely, ZnO at 5%, ZnO at 10%, Ag/ZnO with 0.1% Ag and 10% ZnO, Ag/ZnO with 0.05% Ag and 10% ZnO, Ag/ZnO with 0.1% Ag and 5% ZnO, and Ag/ZnO with 0.05% Ag and 5% of ZnO. Negative controls were wells with composite resin without any nanoparticles and a well without any material to investigate any possible contamination. Positive control was a well with pathogen and culture media. One-way analysis of variance [4] was run to determine any significant differences in width of inhibitory zone of the study groups, followed by high significant difference Tukey test (HSD Tukey) for pair-wise comparisons.

### 2.5. MTT (3-(4,5-Dimethylthiazol-2-yl)-2,5-diphenyl-2H-tetrazolium Bromide) Assay for Cell Viability

HGF (human gingival fibroblast) cells (7 × 10^4^ cells/well) were incubated in 96-well plates, each containing 200 *µ*L of supplemented cell culture media, for 24 hours at 37°C and 5% CO_2_. The cells were divided into 4 groups in triplicates, blank, Z, AZ, and A&Z nanoparticles (different concentrations: 1, 2, 5, 10, and 25 *μ*g/ml), and were treated. After an incubation period of 24 h, the spent media were removed and the plate wells were washed with phosphate-buffered solution. In brief, 50 *μ*L of 2 mg/mL MTT (3-(4,5-dimethylthiazol-2-yl)-2,5-diphenyl-tetrazolium bromide) and 150 *μ*L of culture medium was added to each well. The cells were incubated at 37°C and 5% CO_2_ for 4 hours, and then the media were discarded. Dimethyl sulfoxide and Sorensen buffer were added to each well as solubilizer buffer. Finally, absorbance was read using an ELISA plate reader (BioTek, Bad Friedrichshall, Germany) at 570 nm wavelength.

### 2.6. Wettability Measurements

The wettability of the samples was assessed by measuring the contact angles of distilled water on composite resins with Adobe Photoshop^®^ software. The contact angle was defined as the angle at which the liquid interface met the solid surface of the composite disc at four points on each sample, and the mean of the points was reported as the contact angle of each sample. The surface of the drop was continuously monitored, and the contact angle was measured just after 20 seconds when the droplet was stabilized.

### 2.7. Statistical Analysis

Data were analyzed using Anderson–Darling and Levine tests to check the homoscedasticity and normality, thereof. Standard deviations were calculated for all repeat contact angle measurements and averaged for each series. A one-way ANOVA test was used for data comparison. Tukey's test was used to check the significance of differences between pairs of means. All statistical tests were run at 5% significance level (*P* < 0.05).

## 3. Results

### 3.1. Characteristics Analysis

Figure 1 shows the powder XRD patterns of as-prepared ZnO and Ag/ZnO recorded in the range of 30–70° with a scanning step of 0.02°. The observed diffraction peaks of the pure ZnO catalyst can be indexed to those of hexagonal wurtzite ZnO (PCPDF79-0207). No characteristic peaks of impurity phases such as Zn, Zn(OH)_2_, Ag, or Ag(OH) were observed.

Figure 2 indicates the distribution of nanoparticles in composite resins which demonstrates homogenous disposition of the NPs in the resin matrix.

For the release test, after 30 days' period for composites containing AZ, A&Z, Z nanoparticles, no significant release of silver or zinc ions was detected and the values were zero for both named ions at time intervals of 7, 14, and 30 days.

### 3.2. Shear Bond Strength Test

In this study, 4 different types of orthodontic composite resins were evaluated. In group 1, conventional composite resin (O) was used, and in the other 3 groups, composite resins with ZnO nanoparticles (Z), ZnO and silver nanoparticle solution (A&Z), and Ag/ZnO nanoparticles (AZ) synthesized with optical precipitation were used.

Table 1 presents the descriptive data of shear bond strength tests in each study group separately. Based on these data, the mean shear bond strength value in the A&Z group was lower than that in other groups, with the highest shear bond strength in the AZ group (Figure 3).

The Kolmogorov–Smirnov test showed normal distribution of data in the present study (*P* > 0.05). In addition, Levene's test showed that the variances of the groups were the same (*P* > 0.05). Therefore, one-way ANOVA was used to compare the mean shear bond strength values between the study groups, which revealed significant differences in mean shear bond strength values between the different study groups (*P* = 0.0001). The Tukey test showed that the mean shear bond strength of A&Z composite resin was significantly less than that of conventional composite resin (*P* < 0.05).

### 3.3. Antimicrobial Properties

The results of antimicrobial properties are presented in Table 2. These results include different concentrations of composite with concentrations including ZnO at 5%, ZnO at 10%, Ag/ZnO with 0.1% Ag and 10% ZnO, Ag/ZnO with 0.05% Ag and 10% ZnO, Ag/ZnO with 0.1% Ag and 5% ZnO, and Ag/ZnO with 0.05% Ag and 5% of ZnO, which shows no growth for all Gram-positive pathogens (*P* < 0.05) and slight antimicrobial properties against Gram-negative (*E. coli*) pathogen. In all wells of *C. albicans*, growth was observed. ZnO with 10% concentration had higher antimicrobial properties than 5% concentration.

### 3.4. Viability Test

According to the results obtained from the MTT test, the cytotoxicity of AZ and ZnO nanoparticles indicated that certainly no major and significant damaging effect is expected to the cells up to 0.1 mg/ml of ZnO and AZ nanoparticles. Data are summarized via Figure 4.

### 3.5. Wettability Measurements

The means and standard deviations of the contact angles of the studied groups are summarized in Table 3. The contact angle was not significantly different between the O group and other groups (Z, AZ, and A&Z). Since the contact angles of all groups are less than 90°, both of them are hydrophilic.

## 4. Discussion

Patients' cooperation to observe the oral hygiene has always been a challenge during orthodontic treatment. Many clinicians prefer methods that do not require patient cooperation. Although fluoride-releasing materials are appropriate for patients susceptible to caries, they are predominantly used in the dental office and there are also limitations in relation to the number of times they can be used [14].

The present study was undertaken to evaluate the effect of incorporating nanoparticles into orthodontic composite resins on the antibacterial properties and shear bond strength of these composite resins, which indicated that composite resin with nanoparticles (AZ, A&Z, and Z) had antibacterial properties against oral pathogens. Of all these nanoparticles, AZ nanoparticles synthesized using optical precipitation (AZ composite resin) exhibited antibacterial activity even at lower concentrations (5%), but ZnO nanoparticles (10%) and ZnO nanoparticles containing silver ions exhibited antibacterial activity at higher concentrations (15–20%).

These results indicated the strong antimicrobial properties for these nanocomposites. Most of the nanocomposite resins have better antimicrobial properties for Gram-positive pathogens. The results of the present study showed that these composites had significant antimicrobial properties against *S. mutans*, *S. aureus*, and *L. gasseri* but less power against *E. coli* and no effect against *C. albicans*.

A number of studies have assessed the antibacterial properties of silver nanoparticles [15]. A study by Alt et al. demonstrated the antibacterial activity of silver nanoparticles against resistant pathogens [16]. However, silver nanoparticles induce dark gray discoloration in composite resins, creating problems for dental applications [17]. Eslamian et al. evaluated the effect of Ag nanoparticle (50 nm, 0.3% w/w) incorporation to the conventional orthodontic adhesive to form an orthodontic nanoadhesive. According to results, this nanoadhesive is associated with significant antibacterial properties, which endured for 30 days. Moreover, incorporating AgNPs caused a significant reduction of the mean SBS in the nanoadhesive group [18]. On the other hand, the results of a study by Tavassoli Hojati et al. on the effect of adding ZnO nanoparticles to flowable composite resins on their antibacterial and physical properties and strength showed that an increase in these nanoparticles resulted in a significant increase in their antibacterial activity. In addition, they showed that incorporation of nanoparticles into composite resins resulted in a significant increase in the compressive strength and shear bond strength of composite resins, with no changes in their flexural strength [9]. In our study, although the shear bond strength of AZ nanoparticle-containing composite resins, synthesized using optical precipitation, was higher than that in the control group, the difference was not significant statistically. The average shear bond strength for the different groups in our study ranged from 13.61 to 20.49 MPa (Table 1). An important factor is whether the bond strength of media is within a clinically acceptable range. However, there is no clear consensus regarding what the minimum shear bond strength should be, with some reports suggesting a range of 13–21 MPa and others, 6–8 MPa. The average shear strength of all composites tested in this study was >6 MPa, which is considered by studies to be appropriate for routine clinical use [19]. Therefore, incorporation of nanoparticles to orthodontic composite resins does not result in a change in the mechanical properties of these composite resins.

Moreover, Garcia-Contreras et al. evaluated the effect of incorporating titanium nanoparticles into glass ionomer and concluded that incorporation of these particles increases the compressive and flexural strengths of glass ionomers, in addition to conferring antibacterial properties. In their study, as well, no changes were detected in the shear bond strength to enamel [20]. Poosti et al. showed in another study that incorporation of titanium nanoparticles into orthodontic composite resins confers antibacterial properties, with no changes in the shear bond strength [17]. In another study by Cheng et al. in 2012, incorporation of silver nanoparticles into composite resins improved the mechanical properties of these composite resins and they exhibited antibacterial properties but silver nanoparticles create a dark gray color change in composites, which defies the esthetic purposes [21]. The antibacterial mechanism of ZnO involves its activity as an activator for enzymes. It is toxic to bacteria at a concentration of 0.5 ppm, and concentrations of 4, 6, and 16 ppm can inhibit bacterial growth [13].

Finally, Argueta-Figueroa et al. in 2015 showed that the shear bond strength of orthodontic adhesives, containing copper nanoparticles, was reported to be higher than that in the control group, with no changes in color and other properties [22].

Clinical trials are the ideal methodology for biocompatibility evaluation. Nevertheless, this approach is restricted by ethical considerations. Dental materials must be assessed through several toxicity and biocompatibility steps before being used in the clinic. The definition of biocompatible dental material is to have no or infrequent harmful effects on oral tissue [11]. According to the results obtained from the MTT test, the cytotoxicity of AZ and ZnO nanoparticles indicated that certainly no major and significant damaging effect is expected to the cells up to 0.1 mg/ml of ZnO and AZ nanoparticles. Based on the results of this study, it can be seen that, in the presence of all nanocomposites in the current study, the major bacteria in dental and oral caries (*Streptococcus mutans*, *Lactobacillus*, and *Candida albicans*) cannot grow sufficiently; due to the long presence of orthodontic brackets in the mouth, the formation of plaque and dental caries can be reduced. It should be noted that the release of nanoparticles from polymerized nanocomposites is zero in all three periods of time. In fact, these nanocomposites retain their properties for a long time without delaying the nanoparticles, and because of these unique properties, using these nanoparticles in orthodontic composite resins is suggested. Meanwhile, since the nanocomposites studied are hydrophobic, and as a result, the absorption of bacterial plaques is also reduced, which is a significant advantage in orthodontic use. Lower toxicity and similar tooth coloring of nanoparticles containing zinc oxide with a slight difference in bond strength compared to the control group tend to be more productive for nanocomposites containing this material.

## 5. Conclusion

The present study found that incorporation of different nanoparticles (ZnO, ZnO and silver ions, and Ag/ZnO synthesized) into orthodontic composite resins induced antibacterial properties against oral pathogens. Of all these nanoparticles, AZ exhibited antibacterial activity even at lower concentrations (5%). Based on the MTT cell viability test, the concentration of AZ and ZnO nanoparticles up to 0.1 mg/ml was biocompatible and had no major and significant damaging effect to the human cells. Also, incorporation of AZ into orthodontic composite resins did not change mechanical properties; however, incorporation of ZnO nanoparticles containing silver ions decreased the shear bond strength, but this reduction probably is not concerned clinically.

## Figures and Tables

**Figure 1:** XRD pattern of Ag/ZnO nanoparticles. The existence of high-grade peaks proves the creation of a ZnO system.

**Figure 2:** Zn and Ag map of the resin composite containing 10 wt % Ag/ZnO. Light yellow spots represent Zn, and blue ones represent Ag element.

**Figure 3:** Comparison of shear bond strength in each study group.

**Figure 4:** Effects of the Ag/ZnO and ZnO nanoparticles on cell viability in HGF cells. Data are expressed as the mean of percent cell viability compared to control after exposure for 24 hours ± standard deviation (*n* = 3) (*P* = 0.05).

**Table 1:** The descriptive data of shear bond strength in each study group.

Group	Number	Mean of shear bond strength (MPa)	Std. deviation	Minimum	Maximum
A (O)	30	19.03	4.12	13.42	28.95
B (Z)	30	16.35	1.11	7.90	32.63
C (A&Z)	30	13.61	0.73	8.64	22.61
D (AZ)	30	20.49	1.03	10.48	32.17
Total	120	17.37	0.51	7.90	32.63

Different capital letters indicate different types of orthodontic composite resins, where A (O) stands for conventional composite resin, B (Z) for ZnO nanoparticles, C (A&Z) for ZnO and silver nanoparticle solution, and D (AZ) for Ag/ZnO nanoparticles (*P* < 0.05).

**Table 2:** Antimicrobial effects of the test nanoparticles.

Test groups containing Ag and ZnO (wt %)	Bacteria group (colony-forming unit)				
	*S. mutans* ATCC 35668	*S. aureus* ATCC 25923	*E. coli* ATCC 25922	*C. albicans* ATCC 10231	*Lactobacillus gasseri*
*A*. *ZnO* [10%]	0	0	0	1500	0
*B*. *ZnO* [5%]	0	0	500	50000	0
*C*.*Ag*[0.1%]/*ZnO* [10%]	0	0	0	10000	0
*D*. *Ag*[0.05%]/*ZnO* [10%]	0	0	0	20000	0
*E*. *Ag*[0.1%]/*ZnO* [5%]	0	0	7	50000	0
*F*. *Ag*[0.05%]/*ZnO* [5%]	0	0	32	>10000	0
Control (−)	0	0	0	0	0
Control (+)	>10000	>10000	>10000	>10000	>10000

**Table 3:** The contact angles of the composites in degrees (mean ± SD).

Composite	Contact angle
Conventional composite resin (O)	48.40 ± 2.24
ZnO nanoparticles composite resin (Z)	51.08 ± 1.86
ZnO nanoparticles and silver ions composite resin (A&Z)	54.32 ± 3.54
Ag/ZnO nanoparticles composite resin (AZ)	55.74 ± 5.38

## Data Availability

The data used to support the findings of this study are available from the corresponding author upon request.
